The article "Investigation on Thrust Force Conversion Method of Oscillating Caudal Fin Based on Wake Vortex Field Structure" was published in 2021. Journal: Appl Bionics Biomech.

# Investigation on Thrust Force Conversion Method of Oscillating Caudal Fin Based on Wake Vortex Field Structure

**DOI:** 10.1155/2021/5561268

**Published:** 2021-12-27

**Authors:** Hongjie Ling, Zhidong Wang

**Affiliations:** Jiangsu University of Science and Technology, Zhenjiang 212003, China

## Abstract

The wake field of the flexible oscillating caudal fin is investigated using the Digital Particle Image Velocity (DPIV) system. The distributions of the vorticity with different Strouhal numbers are presented, and a self-developed program is used for calculating the velocity circulation of the vortex ring. Quantitative analysis of the wake field such as velocity circulation of the vortex ring, vortex radius, and the center-to-center spacing of vortex pair is presented. A three-dimensional vortex ring chain model of oscillating caudal fin is introduced. A conversion model between velocity circulation and dynamic moment of the vortex ring is presented according to the vortex dynamics theory, and a self-developed program is used for the calculation, in which the conversion of the thrust force based on wake field of oscillating caudal fin is carried out. Comparisons of the results of the two kinds flexible caudal fins thrust force conversion with the result of tricomponent balance system have been done in this paper. The relative errors are 5.86% and 3.44%, respectively. It is shown that the thrust force conversion model of flexible oscillating caudal fin is accurate and reliable, and the method presented in the paper provides an effective model for the quantitative conversion between the flow field and the thrust force of the caudal fin.

## 1. Introduction

The formation, evolution, and shedding of vortex are controlled by the oscillating of the fish body, and the caudal fin while fish is swimming. Fish whether can get higher thrust force and propulsion efficiency is dominated by the different wake vortex field. The quantitative conversion relationship of the relevant parameters exists between the structural type of the wake vortex field and propulsion performance of the caudal fin. Hence, tests and analysis on the information of vortex field structure of the oscillating caudal fin are needed, and a quantitative conversion model between the information of the flow field and the thrust force of the caudal fin is introduced, which is very important on both exploring the inherent character of fish's high-efficiency swimming and designing a high-efficiency bionic propulsion system.

Gray [1] introduced Gray paradox theory which caused a research boom on propulsion characteristics of fish's high-efficiency swimming. Currently, methods of theoretical analysis, numerical computation, and tests are mainly used to study the structural type of the wake vortex and the wake field of the caudal fin [2–5]. Nguyen et al. [6] used a three-dimensional (3D) Computational Fluid Dynamics (CFD) model to simulate the tail fin motion of a fish robot actuated by a piezoceramic composite actuator and to determine the maximum thrust tail-beat frequency. A simulation of the tail fin at a tail-beat frequency was performed to confirm the measured thrust data from the previous study. The computed and measured thrusts were in good agreement. Lau et al. [7] designed an experiment to study the variation of wake vortex structure generated by hydrofoil's heave-pitch motion with different Strouhal numbers and studied the relationship among the wake vortex structure, the drag force, and the thrust force. The vortex control mechanism of fish-like swimming was investigated by a three-dimensional fish-like model based on nonlinear inviscid numerical method (Zhu et al. [8]). Wang and Zhang [9, 10] studied the evolution character of the wake vortex of the oscillating caudal fin and the effect of the chordwise and spanwise deformation on wake vortex structure.

The article "Investigation on Thrust Force Conversion Method of Oscillating Caudal Fin Based on Wake Vortex Field Structure" was published in 2021. Journal: Appl Bionics Biomech.

Yang et al. **[**11**]** used DPIV to measure the velocity and vorticity fields generated by a thin circular disk, and the finite-time Lyapunov exponent field corresponding to the vortex flow was computed to identify Lagrangian coherent structures of the starting vortex. Nauen et al. [12] used DPIV to test the wake structure at different areas of the homocercal caudal fin of the euthynnus and compared the thrust force with the drag force at the same speed. Maneuverability characteristics under different propulsion efficiencies were introduced. By testing the vertical light sheet, moment balance relationship of the lift force provided by caudal fin and pectoral fin to the center of mass was obtained. Tangorra et al. [13] studied the pectoral fin of the bluegill sunfish based on the theory of anatomy, kinematics, and hydrodynamics and designed a sunfish-like pectoral fin propeller. Thrust force generated by pectoral fin under different working conditions was obtained by CFD simulation and hydrodynamic tests, and the effect of the amplitude of the oscillation and the crimp on thrust force was investigated. Drucker and Lauder [14] used the DPIV system to test the three-dimensional flow field of the bluegill sunfish and presented a 3D vortex ring according to the information of flow field. Thrust force, lift force, and drag force generated by the oscillation of the pectoral fins were obtained by the conversion, and the reacting force of fluid acted on the pectoral fins was obtained according to the direction of vortex ring and jet flow. It is shown that DPIV technology could be adopted to test the flow field of complex vortex and unsteady flow. The conversion model between the wake vortex and thrust force of fish body was presented. Sakakibara et al. [15] used DPIV to measure the three-component velocity distribution around a live fish. The thrust force and time-averaged force excited by oscillating caudal fin were evaluated based on the 3D vortex ring which was generated by measured flow field information. Li et al. [16] used DPIV to study the wake flow field of live fish and presented the reversed Karman vortex street and vortex ring model.

The article "Investigation on Thrust Force Conversion Method of Oscillating Caudal Fin Based on Wake Vortex Field Structure" was published in 2021. Journal: Appl Bionics Biomech.

In this paper, tests on the flow field of the oscillating caudal fin are conducted using the DPIV system. A computational program is developed based on the information of velocity field which is obtained by the test. Quantitative information such as velocity circulation and radius of vortex ring in wake vortex filed are obtained, and then, a conversion model between the velocity circulation and the dynamic moment of the vortex ring is presented using the Kelvin theory, and a self-developed program is used for the calculation in which the quantitative analysis of the wake vortex field structure, and conversion of the thrust force of the caudal fin is carried out. Methods presented in this paper provided an accurate and reliable method for the comprehensive analysis on the quantitative relationship among the oscillation parameters, the information of the flow field, and the propulsion character of the caudal fin.

## 2. Experimental Equipment and Parameter Setting

The experimental equipment includes two flexible caudal fins, the system of DPIV, caudal fin drive, and tricomponent balance. In Figure 1, the flexible caudal fin is made of rubber material. The measured modulus of elasticity is 7.8 MPa according to the GB/T 1040-92 specification, the drive system is shown in Figure 2, and the general arrangement of experimental system is shown in Figure 3. The control system consists of the optical electric axial angle encoder and the programmable logic controller. In order to combine the signal control of the shooting of the flow field and the oscillating angle of the caudal fin during the experiment, a synchronous control program is developed based on the optical electric axial angle encoder and the programmable logic controller, the real-time synchronous control of the oscillating angle of caudal fin, and the flow field shooting are carried out.

The equation of the oscillating caudal fin is given as follows:

(1) $$\begin{array}{c} \theta \left(t\right)=\theta_{\max}\cos\left(4.16\pi t+\frac{\pi }{2}\right), \end{array}$$

where *θ*_max_ is the amplitude of the oscillation of the caudal fin, the Strouhal number is defined as St = *fh*/*v*, where *h* is the width of the wake vortex, in general, *h* approximately sets to the maximum amplitude of the oscillation on the rear edge of the caudal fin, *f* denotes the frequency of the caudal fin oscillation in Hz, and *v* is the velocity of water flow.

The article "Investigation on Thrust Force Conversion Method of Oscillating Caudal Fin Based on Wake Vortex Field Structure" was published in 2021. Journal: Appl Bionics Biomech.

## 3. Wake Vortex Field of Oscillating Caudal Fin

Tests on the flow field of the oscillating caudal fin are carried out with four different Strouhal numbers: St =0.39, 0.43, 0.54, and 0.6. Corresponding vorticity field distribution graphs are presented in Figure 4 (the unit of horizontal and vertical coordinates is mm, and the unit of vorticity is s^−1^). The red vortex means the vorticity number is positive, and the blue vortex means the vorticity number is negative, which are referred to as the positive vorticity and negative vorticity, respectively. Vorticity number increases with the increment of Strouhal number and the center-to-center spacing between the positive vorticity, and the negative vorticity is the diameter of the vortex ring.

## 4. Calculation Method for Velocity Circulation of Vortex Pair and 3D Vortex Ring Chain Model

In order to calculate the geometry size of vortex in the wake field, the radius of the vortex needs to be defined. Based on the corresponding velocity, circulations of the vortex surrounded by different integration paths are same, we choose the vortex center as origin, a series of closed contours are constructed with circles of different radii, and these closed contours are used as integration path for the calculation of corresponding velocity circulation.

Take the relative coordinate system oxy, take 8 points uniformly along the circumference, and the center angles of the circle are as follows: 0, *π*/4, *π*/2, 3*π*/4, *π*, 5*π*/4, 3*π*/4, and 7*π*/4.

The velocity at any point on the circumference is $\overset{⟶}{V}$, and the velocity decomposition is shown in Figure 5.

Figure 6 shows the following:

(2) $$\begin{array}{c} dx=dl\cdot \cos\;\theta , \end{array}$$

(3) $$\begin{array}{c} dy=dl\cdot \sin\;\theta , \end{array}$$

(4) $$\begin{array}{c} dl=Rd\theta . \end{array}$$

The formula of the velocity circulation is given as follows:

(5) $$\begin{array}{c} \Gamma =\int \overset{⟶}{V}\cdot dl=\int V_{x}dx+V_{y}dy=\int V_{x}\cos\;\theta dl+V_{y}\sin\;\theta dl=\int \left(V_{x}\cos\;\theta +V_{y}\sin\;\theta \right)Rd\theta , \end{array}$$

where $\overset{⟶}{v}$ is the tangential component of the velocity vector, *dl* is integration path, and the radius is the same with the vortex radius when the velocity circulation is to maximum value. It is assumed that in each interval, *V*_*x*_ and *v*_*y*_ change linearly. Let *n* ∈ (0, 7) be the interval range, and *θ* is expressed in radians. For a point (*x*, *y*) in any interval, the following formula is satisfied:

(6) $$\begin{array}{c} \int_{\left(n-1\right)\pi /4}^{n\pi /4}\overset{⟶}{V}\cdot dl=\int_{\left(n-1\right)\pi /4}^{n\pi /4}\left(V_{x}\cos\;\theta +V_{y}\sin\;\theta \right)Rd\theta =\int_{\left(n-1\right)\pi /4}^{n\pi /4}\left[\left(V_{xn}+\left(\frac{4\theta }{\pi }-n\right)\left(V_{xn+1}-V_{xn}\right)\right)\cos\left(\theta -\frac{\pi }{4}n\right)\right.. \end{array}$$

The derived calculation formula of velocity circulation is as follows:

(7) $$\begin{array}{c} \Gamma =\int \overset{⟶}{V}\cdot dl=\overset{7}{\underset{n=0}{\sum }}\int_{n\pi /4}^{\left(n+1\right)\pi /4}\left[\left(V_{xn}+\left(\frac{4\theta }{\pi }-n\right)\left(V_{xn+1}-V_{xn}\right)\right)\cos\left(\theta -\frac{\pi }{4}n\right)\right.\left.+\left(V_{yn}+\left(\frac{4\theta }{\pi }-n\right)\left(V_{yn+1}-V_{yn}\right)\right)\sin\left(\theta -\frac{\pi }{4}n\right)\right]\cdot R\cdot d\theta , \end{array}$$

where *n* ∈ [0, 7] represents eight intervals divided on the contour and *V*_*nx*_ and *V*_*ny*_ are the velocity components on the discrete points. Integration path of wake vortex velocity circulation is shown in Figure 7.

The article "Investigation on Thrust Force Conversion Method of Oscillating Caudal Fin Based on Wake Vortex Field Structure" was published in 2021. Journal: Appl Bionics Biomech.

The two-dimensional vortex on a plane is actually corresponded to a three-dimensional vortex ring according to vortex dynamics theory. Radii of the wake vortex and vortex ring generated by oscillating caudal fin under the test are obtained by the calculation of the velocity circulation and the center-to-center spacing of the vortex pair in the wake flow field. And the three-dimensional structure of the vortex ring of the oscillating caudal fin flow field is presented, which is shown in Figures 8 and 9.

## 5. Conversion of Flow Field Structure and Caudal Fin Thrust Force

According to Kelvin's theorem (vortex dynamics theory), thrust force of the oscillating caudal fin can be obtained by velocity circulation Γ in the wake vortex field. Dickinson and Gotz [17] further point out that the reaction force acted on the oscillating hydrofoil is supplied by the shed vortex ring momentum in the wake vortex field. The momentum (*M*) of a vortex ring shed into the wake is estimated using *M* = *ρ*Γ*A*, where *ρ* is the water density, Γ is the velocity circulation, and *A* is the projected area of the vortex ring. Γ and *A* are measured at the end of the fin-oscillating cycle. The corresponding instantaneous dynamic force and time-averaged dynamic force of the vortex ring are, respectively, given as follows:

(8) $$\begin{array}{c} F=\frac{dM}{dt}, \end{array}$$

(9) $$\begin{array}{c} \bar{F}=\frac{\rho \Gamma A}{T}. \end{array}$$

In the paper, the time-averaged thrust force generated by the momentum of the shed vortex ring is calculated according to the vortex dynamics theorem. As the angle between the connecting lines of the vortex centers and the opposite direction of the water flow is *α*, as shown in Figure 10, the thrust force and lateral force generated by time-averaged dynamic force are given, respectively, as follows:

(10) $$\begin{array}{c} F_{1}=\bar{F}\cdot \sin\alpha , \end{array}$$

(11) $$\begin{array}{c} F_{2}=\bar{F}\cdot \cos\alpha . \end{array}$$

Using C++ language, a calculation program was written to solve formulas (2)–(11) to realize the conversion of vortex ring velocity, torque, and thrust. The thrust and torque can be automatically calculated based on the DPIV test flow field information.

The article "Investigation on Thrust Force Conversion Method of Oscillating Caudal Fin Based on Wake Vortex Field Structure" was published in 2021. Journal: Appl Bionics Biomech.

In the paper, the tests of the two kinds of flexible caudal fins (elastic modulus are *E*1 = 4.3 MPa, *E*2 = 7.8 MPa) with the flow speed *v* = 0.176 m/s and the caudal fin oscillating frequency *f* = 0.91 Hz are carried out in the wake vortex field for the thrust force conversion, while the thrust force of the flexible caudal fins using tri-component balance [18] is measured.  Table 1 shows the comparison of the testing result with the theoretical conversion result, and the relative errors of the results of the two kinds flexible caudal fins thrust conversion and the testing result of tricomponent balance are 5.86% and 3.44%, respectively. It is shown that the present thrust conversion model of flexible oscillating caudal fin is accurate, the results are reliable, and it can be used in the study of high-efficiency propulsion mechanism of fish's caudal fin.

## 6. Conclusion

In this paper, tests on the flow field of the oscillating caudal fin are carried out based on the DPIV system. Vorticity field distributions with different Strouhal numbers are presented, and a self-developed program is used for the calculation of the velocity circulation of the vortex ring. Basic information of the wake field such as velocity circulation and the radius of the vortex ring are obtained. A three-dimensional vortex ring chain model of the oscillating caudal fin is introduced, and the calculation principles of the velocity circulation, vortex dynamic moment, and the thrust force of caudal fin are theoretically analyzed, and a self-developed program is used in the conversional computation on the velocity circulation of the wake vortex and the vortex dynamic moment of the oscillating caudal fin in which the quantitative conversion based on the information of the flow field and the thrust force of the caudal fin is presented. And the numerical results are compared with the test results in this paper. It is shown that methods occupied in this paper provide an effective method for the quantitative analysis between the flow field structure and the thrust force performance of the caudal fin.

The article "Investigation on Thrust Force Conversion Method of Oscillating Caudal Fin Based on Wake Vortex Field Structure" was published in 2021. Journal: Appl Bionics Biomech.

## Figures and Tables

**Figure 1:** Flexible caudal fin model.

**Figure 2:** Caudal fin drive system.

**Figure 3:** Water tank and equipment arrangement.

**Figure 4:** Vorticity field of flexible oscillating caudal fin with different Strouhal numbers.

**Figure 5:** Velocity resolution and component expression.

**Figure 6:** Relation between the arc length and radius.

**Figure 7:** Integration path of wake vortex velocity circulation.

**Figure 8:** Vortex radius and vortex ring radius.

**Figure 9:** 3D vortex ring model of oscillating caudal fin.

**Figure 10:** Time-averaged thrust force and lateral component.

**Table 1:** Comparison on numerical conversion in this paper and experimental results in literature of caudal fin thrust force.

Model	Flexible caudal fin *E*1 = 4.3 MPa	Flexible caudal fin *E*2 = 7.8 MPa
Experimental condition (1)	*v* = 0.176 m/s *f* = 0.91 Hz	*v* = 0.176 m/s *f* = 0.91 Hz
Theoretical results (mN)	51.39	44.85
Measurement results (mN)	48.38	43.31
Error	5.86%	3.44%

## Data Availability

The experimental data used to support the findings of this study are included within the article.
